# Transcription elongation factor A-like 7, regulated by miR-758-3p inhibits the progression of melanoma through decreasing the expression levels of c-Myc and AKT1

This article has been retracted.

**DOI:** 10.1186/s12935-020-01737-3

**Published:** 2021-01-11

**Authors:** Xilin Liu, Xianji Song, Hong Li

**Affiliations:** 1 Department of Hand Surgery, China Japan Union Hospital of Jilin University, Changchun, 130033 Jilin China; 2 Orthopaedic Surgery, China Japan Union Hospital of Jilin University, Changchun, 130033 Jilin China; 3 Emergency Medical of China Japan Union Hospital of Jilin University, No. 126 Xian Tai Street, Changchun, 130033 Jilin China

**Keywords:** Melanoma, miR-758-3p, TCEAL7, Cell function, Tumorigenesis

## Abstract

**Background:**

Ectopic expression of transcription elongation factor A (SII)-like 7 (TCEAL7) has been observed in several kinds of cancers, but its role in melanoma is still unclear. This study was carried out to investigate TCEAL7 role in melanoma progression, and uncover the underlying mechanisms.

**Methods:**

TCEAL7 expression levels in melanoma tissues and cells were determined by using real-time quantitative PCR (RT-PCR) and western blotting. CCK-8, transwell chambers, flow cytometry, starch assay and tumorigenesis assay were applied to detect cell growth, invasion, apoptosis, migration and tumorigenesis, respectively.

**Results:**

A low expression level of TCEAL7 was observed in melanoma tissues and cells, which was associated with malignant clinical process and poor prognosis. TCEAL7 negatively modulated AKT1, AKT2, c-Myc, N-cadherin and PCNA expression and inhibited cancer progression via decreasing AKT1 and c-Myc levels. In addition, TCEAL7 was negatively modulated by miR-758-3p which promoted melanoma progression. Moreover, overexpression of TCEAL7 abolished miR-758-3p role in promoting melanoma progression.

**Conclusion:**

This study demonstrated that TCEAL7, regulated by miR-758-3p inhibited melanoma progression through decreasing the expression levels of c-Myc and AKT1.

## Introduction

Melanoma, as a type of skin cancer, is a malignant tumor with a high metastatic potential [1, 2]. According to the most recent data in Cancer Genomics Consortium (http://www.cancergenomics.org/), the 5-year overall survival rate for primary melanoma is 92%. However, the 5-year survival rate for metastatic melanoma is only 25%. Thus, further explorations of the molecular mechanisms underlying the progression of malignant melanoma are desperately needed.

Transcription elongation factor A (SII)-like 7 (TCEAL7) encodes a cell death regulatory protein, which is inactivated by methylation [3] and has a sequence similarity to brain-expressed (Bex) proteins, TCEAL1 and TCEAL6 [4, 5]. TCEAL7 has been identified to be frequently deregulated in tumors, and its decreased expression often correlates with malignant clinical process and poor prognosis in several kinds of cancers, such as ovarian cancer [4], gastric adenocarcinoma [6] and non-small cell lung cancer [7]. Re-expression of TCEAL7 in ovarian cancer cell lines (OV 167, OV 177, OV 202, OV 207, OV 266, OVCAR-5 and SKOV-3) induces cell death and inhibits cell colony formation efficiency [4]. Knockdown of TCEAL7 increases the activity of oncogenic gene c-Myc in epithelial ovarian cancer cell lines [8]. Downregulation of TCEAL7 enhances the expression levels of proliferative, angiogenic, inflammatory and anti-apoptotic genes in ovarian cancer cells through the nuclear factor kappa B (NF-κB) pathway [3]. All of these findings suggest that TCEAL7 serves as a tumor suppressor in ovarian cancer. However, TCEAL7 function in malignant melanoma still needs to be uncovered.

Increasing evidence demonstrates that microRNAs (miRNAs) are strongly implicated in tumorigenesis via degradation and/or translational suppression of mRNAs through binding to the 3′‑untranslated regions (UTRs) of the target genes [9, 10]. miR-758 was found to be lowly expressed in retinoblastoma tissues and cell lines, and restoration of its expression caused significant inhibitions in cell proliferation, invasion and migration capacities, and increased cell apoptosis via targeting paired box protein 6 (PAX6) [11]. It is predicted that TCEAL7 is a target of miR-758-3p using the online software miRanda and miRDB. However, whether miR-758-3p is involved in the progression of melanoma via targeting TCEAL7 remains unknown.

In this paper, we aimed to explore the role of TCEAL7 in the progression of melanoma and uncover whether miR-758-3p targets TCEAL7 to participate in melanoma progression.

## Materials and methods

### Bioinformatics analysis

TCEAL7 expression levels in melanoma tissues and normal tissues were analyzed by using the Gene Expression Profiling Interactive Analysis (GEPIA; http://gepia.cancer-pku.cn/). The correlations between the levels of TCEAL7, AKT1, AKT2 and c-Myc were analyzed by using the starBase (http://starbase.sysu.edu.cn/). The miRanda (http://microrna.org/microrna/home.do) and miRDB (http://www.mirdb.org/index.html) [12–14] were applied to predict the miRNAs which target TCEAL7.

### Patients and sample preparation

Ninety-eight fresh melanoma tissues were obtained from patients with melanoma. Thirty nevus tissues (benign proliferation of melanocytes) obtained from age and gender-matched individuals served as normal control. None of interventional treatment was performed before surgery.

### Cell culture

A375, one human malignant melanoma cell line was purchased from the Cell Bank of the Chinese Academy of Sciences (Shanghai, China); WM-115, another human melanoma cell line and the normal melanocytes PIG1 were purchased from American Type Culture Collection (ATCC, Manassas, VA, USA). All cells were cultured in DMEM (Hyclone, USA) with 10% fetal bovine serum (FBS) (Hyclone) in a humidified incubator at 37 °C with 5% CO_2_.

### RNA interference and lentivirus construction

The small interfering RNAs (siRNAs) targeting the human TCEAL7 gene were designed and synthesized by the GenePharma Co., LTD (Sghanghai, China). The sequences are listed as follows:

si-TCEAL7-1: 5′-CCGAAGTCCTTATATTCCCGGGCTT-3′;

si-TCEAL7-2: 5′-GAGCTGACGTGAACCGAAGTCCTTA-3′;

si-TCEAL7-3: 5′-CCAGTCATTCGATGTTGCTGAGATT-3′;

si-Scramble: 5′-CATCAATTGAACCGAGCCTTACGTA-3′. The three siRNAs-TCEAL7 and si-Scramble were transfected into cells by using the Lipofectamine 2000 (Invitrogen, Carlsbad, CA, USA) according to the manufacturer’s instructions.

To upregulate TCEAL7 (Lenti-TCEAL7), miR-758-3p (mimics), AKT1 (Lenti-AKT1) and c-Myc (Lenti-c-Myc) in melanoma cells, the lentivirus vectors were constructed by GenePharma Co., LTD and infected into cells with the help of polybrene (Thermo Fisher Scientific, MA, USA). The infected cells were then probed with 6 μg/ml puromycin and/or 100 μg/ml G418 for 14 days to establish the stably transfected cells, which were used in the in vivo experiments.

### Real-time quantitative PCR (RT-PCR) analysis of mRNA levels

Total RNA isolation from tissues and cells was carried out with the help of Trizol reagent (Invitrogen), which was then reversely transcribed into cDNA using RT^2^ First Strand Kit (Qiagen, Germany) in the light of manufacturer’s instructions. Then, the mRNA levels were assayed by RT-PCR with TransStart Green qPCR SuperMix (TransGen, Beijing, China) in a DA7500 Real-time Nucleic Acid Amplification Fluorescence Detection System (Bio-Rad, USA). GAPDH (glyceraldehyde-3-phosphate dehydrogenase) level was used to normalize the mRNA levels. The 2^−△△Ct^ method was used to calculate the changes of relative mRNA [15]. The experiments were carried out in three replicates. The primers were synthesized by Sangon (Shanghai, China) and listed in Table 1.

**Table 1:** Primer sequences

Gene	Forward (5ʹ-3ʹ)	Reverse (5ʹ-3ʹ)
Homo-TCEAL7	GAGCTGACGTGAACCGAAGT	GGAGGAAGGAGCTATCTGTGG
AKT1	GAAGACGGGAGCAGGCG	TGTACTCCCCTCGTTTGTGC
AKT2	CTGCCACCATGAATGAGGTGAA	CATGGTCACTTTAGCCCGTG
STAT3	CTGTGGGAAGAATCACGCCT	ACATCCTGAAGGTGCTGCTC
β-catenin	CTGAGGAGCAGCTTCAGTCC	GGCCATGTCCAACTCCATCA
TGF-β	GGGCTACCATGCCAACTTCT	GACACAGAGATCCGCAGTCC
YAP	CCCTCGTTTTGCCATGAACC	GTTGCTGCTGGTTGGAGTTG
c-Myc	GCAATGCGTTGCTGGGTTAT	CGCATCCTTGTCCTGTGAGT
FOXO1	TTGAACCCACACGGTGGTAG	CCTCGGCCTCTGAAACACTT
GAPDH	TGCACCACCAACTGCTTAGC	GGCATGGACTGTGGTCATGAG
Mus-TCEAL7	AGGGCTCTGCATTCTAACCG	TCACTGCTTTCCTAACGCGA
AKT1	CCGCCTGATCAAGTTCTCCT	CAGACCCATGAGCCCACATT
AKT2	GTGGCTGGAAAAGGCGGTAT	TTCACACGCTGTCACCTAGC
c-Myc	GTTGGAAACCCCGCAGACAG	GTAGCGACCGCAACATAGGA
GAPDH	AGAGAGGCCCAGCTACTCG	CAAATCCGTTCACACCGACC
miR-758	ACACTCCAGCTGGGAACGATG	CTCAACTGGTGTCGTGGAGTCGGCA
U6	CTCGCTTCGGCAGCACA	AACGCT TCACGAATTTGCGT

### RT-PCR analysis of miRNA levels

The level miR-758-3p was detected by RT-PCR according to a previous study [16]. Briefly, total miRNAs were isolated from tumor samples and cell lines based on the manufacturer's protocol of the miRcute miRNA Isolation kit (Tiangen Biotech Co., Ltd, Beijing, China). After that, the cDNA was synthesized using the miRcute miRNA cDNA kit (Tiangen Biotech Co., Ltd.), and miR-758-3p level was then detected by the miRcute miRNA luciferase quantitative kit (Tiangen Biotech Co., Ltd). U6 was used as an internal reference. The primer sequences were listed in Table 1.

### Western blotting analysis

Total proteins from cells and tissues were obtained with RIPA buffer (Thermo Fisher Scientific) containing protease inhibitor cocktail. Then, the protein concentrations were determined by using the BCA Protein Assay Kit (Thermo Fisher Scientific) based on the instructions. After that, equal amounts of proteins were separated using 10% SDS-PAGE gels and then transferred to the polyvinylidene fluoride membranes (PVDF; Millipore, Dallas, Tx, USA). Next, the 5% skim milk was used to block the PVDF membranes, which was then incubated with the primary antibodies overnight at 4 °C, including TCEAL7 (cat no. 11218-1-AP, Proteintech, Wuhan, China), AKT1 (cat no. ab235958, Abcam, Cambridge, MA, USA), AKT2 (cat no. ab175354, Abcam), p-AKT (cat no. 4060, Cell Signaling Technology, MA, USA), c-Myc (cat no. ab32072, Abcam), STAT3 (cat no. ab68153, Abcam), β-catenin (cat no. ab16051, Abcam), TGF-β (cat no. ab179695, Abcam), p-SMAD2 (cat no. 18338, Cell Signaling Technology), p-SMAD3 (cat no. 9520, Cell Signaling Technology), YAP (cat no. ab52771, Abcam), FOXO1 (cat no. ab52857, Abcam), PCNA (proliferating cell nuclear antigen) (cat no. ab92552, Abcam), E-cadherin (cat no. 14472, Cell Signaling Technology), N-cadherin (cat no. 4061, Cell Signaling Technology) and GAPDH (cat no. 60004-1-Ig, Proteintech). Following incubation with the secondary antibodies for 1 h at room temperature, western blotting luminol reagent (Millipore) was used to visualize the immunoreactive bands.

### Cell proliferation assay

Cell proliferation viability was detected by Cell Counting Kit-8 (CCK-8, Dojindo, Japan) according to the manufacturer’s instructions. In brief, 2 × 10^3^ A375 and WM-115 cells were seeded into 96-well plates overnight prior to transfection/infection. Next, 10 μl of CCK-8 reagent and 90 μl cell culture medium were added into each well after 1, 2, 3, 4 or 5 days of cell transfection/infection, respectively. Following incubation for 2 h at 37 °C with 5% CO_2_, the absorbance of each well was measured at 450 nm.

### Apoptosis assay

The melanoma A375 and WM-115 cells were placed into 6-well plates at a concentration of 5 × 10^5^/well and allowed to grow at 37 °C overnight, followed by cell transfections/infections. After 48 h, the cells were collected for apoptosis detection using Annexin-V-(FITC) and propidium iodide (PI) kit (BD Biosciences, San Jose, CA, USA). The double-stained cells were subsequently analyzed by the BD flow cytometer. At least 1 × 10^5^ cells were detected each time.

### Scratch assay

Melanoma cells were placed in 6-well plates with adequate numbers to reach 100% confluence in the next day. Then, the wounds were made by using 20 μl pipette tips. The non-adherent cells were removed by washing with PBS slowly. After that, each well was added 2 ml culture medium containing 1% FBS. The wound width was measured at 0 and 24 h post the scratch.

### Transwell chamber assay

To assess cell invasion, melanoma cells were suspended in FBS-free DMEM and then inoculated in the Matrigel pre-coated transwell chamber (BD Bioscience), with 1 × 10^5^ cells for each well. The lower chamber was added 600 μl of 10% FBS-DMEM. At 24 h post incubation, the non-invaded cells were removed with cotton swabs, and the invaded cells in the lower surface were fixed with cold 100% methanol and stained with 0.1% crystal violet (Solarbio Co., Ltd, Beijing, China) for 8 min. Pictures were taken under a microscope with a magnification of 200×, and the invaded cells were counted. Five randomly selected fields were recorded for each well.

### Dual luciferase gene reporter assay

Wide type (WT) and mutative type (MUT) of the 3′UTR of TCEAL7 with the putative miR-758-3p-binding sites were chemically synthesized and cloned into the Renilla luciferase gene (pLUC-REPORT vector; Promega, Madison, WI, USA). WM-115 and A375 cells were co-transfected with 200 ng luciferase reporter vector and 100 nM miR-758-3p mimics or the negative controls. Luciferase activity was examined 48 h after the transfection using the Dual-Luciferase Assay kit (Promega) according to manufacturer’s instructions.

### In vivo tumorigenesis assay

The animal experiment was approved by Animal Ethics Committee of China Japan Union Hospital of Jilin University. SPF grade male BALB/c nude mice (6-week-old) were purchased from the Institute of Zoology, Chinese Academy of Sciences. The malignant melanoma cells A375 were re-suspended in 0.1 ml of PBS and subcutaneously injected into 6-week-old male nude mice (2 × 10^6^ cells/mouse). The mice were euthanized 28 days after injection, and the tumors were taken out and weighed.

### Statistical analysis

All statistical analyses were performed by SPSS 19.0 software package (SPSS Inc., Chicago, IL, USA). Data from each group were expressed as mean ± standard error. Overall survival curves were calculated with the Kaplan–Meier method and were analyzed with the log-rank test. Student’s *t* tests and one-way analysis of variance followed by Tukey’s post hoc tests were conducted to analyze differences between 2 and ≥ 3 groups, and *P* < 0.05 was thought as statistical significance.

## Results

### TCEAL7 is downregulated in human melanoma tissues and cell lines

To determine the effects of TCEAL7 on the progression of melanoma, we first analyzed TCEAL7 expression pattern in melanoma with the help of GEPIA database. In comparison with the normal group, TCEAL7 expression level was decreased in melanoma group (Fig. 1a). To verify it, we also explored the expression levels of TCEAL7 in melanoma tissues and cell lines using RT-PCR and western blotting. As shown in Fig. 1b, c, both of the mRNA and protein levels of TCEAL7 in melanoma tissues were obviously decreased as compared with that of the nevus tissues (normal control). In addition, we detected the mRNA and protein levels of TCEAL7 in human normal skin cell line PIG1 and melanoma cell lines, including A375 and WM-115. From the results, we found that the expression level of TCEAL7 was decreased dramatically in malignant melanoma cell line A375 as compared with PIG1, with null in WM-115 cells (Fig. 1d, e). These data demonstrated that TCEAL7 was lowly expressed in melanoma tissues and cell lines, suggesting that TCEAL7 might play an important role in the progression of melanoma.

**Fig. 1:** Analysis of the expression patterns and clinical significance of TCEAL7 in melanoma. **a** GEPIA database was applied to analyze the expression level of TCEAL7 in melanoma tissues and normal tissues. **b**, **c** The expression levels of TCEAL7 in melanoma tissues and nevus tissues at mRNA and protein levels were determined by using RT-PCR and western blotting assays, respectively. **d**, **e**. RT-PCR and western blotting were performed to detect the mRNA and protein levels of TCEAL7 in normal melanocyte cell line PIG1 and melanoma cell lines WM-115 and A375. **f** Kaplan–Meier was used to analyze the prognostic value of TCEAL7 in melanoma patients. (**P < 0.01, ***P < 0.001)

### Clinical significance of TCEAL7 in melanoma

Next, we explored the relationship between the expression levels of TCEAL7 and the clinicopathologic features and prognosis of melanoma patients. As shown in Table 2, the expression level of TCEAL7 showed a negative correlation with the tumor size, histological grade and TNM stage in melanoma patients. The overall survival time of patients with low expression of TCEAL7 was shorter than that of patients with TCEAL7 high expression (Fig. 1f). These results indicated that low expression of TCEAL7 was closely associated with the advanced process and poor prognosis in melanoma patients.

**Table 2:** Association of TCEAL7 expression with clinicopathological features of melanoma patients

Variables	Number (n=98)	TCEAL7 expression		*P* value
		Low (n=55)	High (n=43)	
Age (years)				0.897
< 60	38	21	17	
≥ 60	60	34	26	
Gender				0.997
Male	57	32	25	
Female	41	23	18	
Tumor size (cm)				0.009
≤ 3.0	61	28	33	
> 3.0	37	27	10	
Histological grade				0.011
G1/G2	45	19	26	
G3	53	36	17	
TNM				0.017
I–II	35	14	21	
III–IV	63	41	22	

### TCEAL7 inhibits melanoma cell proliferation, migration and invasion abilities

Then, we explored the effects of TCEAL7 on the progression of melanoma in vitro. TCEAL7 was upregulated in WM-115 and A375 cells, and downregulated in A375 cells. The expressions of TCEAL7 at both mRNA and protein levels in Lenti-TCEAL7 group were increased obviously when compared with the Lenti- NC group, and decreased in the si-TCEAL7-1/-2/-3 transfected cells as compared with the si-NC group (Fig. 2a–f). As si-TCEAL-1 showed the highest knockdown efficiency between the 3 siRNAs of TCEAL7, si-TCEAL7-1 was applied in the following experiments. Next, we determined the effects of TCEAL7 on cell proliferation, invasion, apoptosis and migration abilities using CCK-8, transwell chambers, flow cytometry and scratch assays, respectively. The results showed that cell growth (Fig. 2g, h), invasion (Fig. 2i, j) and migration (Fig. 2m, n) abilities were significantly weakened in Lenti-TCEAL7 group when compared with the Lenti-NC group, and enhanced in si-TCEAL7 group in comparison with the si-NC group. Additionally, we tested the role of TCEAL7 in cell apoptosis by using the flow cytometry technology. Overexpression of TCEAL7 induced cell apoptosis in both WM-115 and A375 cell lines, and knockdown of TCEAL7 resulted in apoptosis inhibition (Fig. 2k, l). Moreover, overexpression of TCEAL7 reduced the expression levels of PCNA (proliferation marker) and N-cadherin (mesenchymal cell marker), and increased E-cadherin (epithelial cell marker) level, while silencing of TCEAL7 caused the opposite results (Fig. 2o, p). These results suggested that TCEAL7 functioned as a tumor suppressor in melanoma.

**Fig. 2:** TCEAL7 inhibited melanoma cell proliferation, invasion and migration, and induced cell apoptosis. **a**–**f** RT-PCR and western blotting assays were used to detect the knockdown and overexpression efficiencies of TCEAL7 in A375 and WM-115 cell lines. **g**, **h** CCK-8 assay was used to test cell proliferation following TCEAL7 was overexpressed/silenced in WM-115 and A375 cells. **i**, **j** Transwell chamber assay was used to test cell invasion ability following TCEAL7 was overexpressed/silenced in WM-115 and A375 cells. **k**, **l** TCEAL7 effect on the apoptosis of WM-115 and A375 cells were detected by flow cytometry. **m**, **n** Starch assay was used to test cell migration ability following TCEAL7 was overexpressed/silenced in WM-115 and A375 cells. **o**, **p** Western blotting assay was used to measure the expression levels of E-cadherin, N-cadherin and PCNA following TCEAL7 was overexpressed/silenced in WM-115 and A375 cells. (*P < 0.05 and **P < 0.01, compared with Lenti-NC group; ^#^*P* < 0.05, compared with si-Scramble group)

### TCEAL7 negatively regulates AKT1, AKT2 and c-Myc expression

To reveal the molecular mechanisms by which TCEAL7 inhibits the progression of melanoma, we explored the effects of TCEAL7 on the expression of key proteins of signaling pathways. Compared with the lenti-NC group, the expression levels of AKT1, AKT2, p-AKT and c-Myc were significantly decreased following TCEAL7 overexpression in WM-115 and A375 cells at mRNA and/or protein levels (Fig. 3a–d), with no obvious change in the expression levels of STAT3, β-catenin, TGF-β, YAP, FOXO1, p-SMAD2 and p-SMAD3. To further clarify the relationship between TCEAL7 and AKT1, AKT2 and c-Myc, the starBase online software was applied to analyze the correlations between the levels of TCEAL7 and AKT1, AKT2 and c-Myc in skin cutaneous melanoma (SKCM). The results showed that TCEAL7 level was negatively correlated with AKT1, AKT2 and c-Myc levels in SKCM samples, with significances for AKT1, AKT2 and c-Myc (Fig. 3e–g). To verify it, we then analysis their correlations in melanoma tissues. However, the Pearson analysis showed that TCEAL7 level was only significantly negatively correlated with AKT1 and c-Myc levels in melanoma samples, with no significant correlation with AKT2 level (Fig. 3h–j). These results illustrated that AKT1 and c-Myc may play a role in TCEAL7-mediated inhibition in melanoma progression.

**Fig. 3:** TCEAL7 increased the expression levels of AKT1, AKT2 and c-Myc in melanoma cells. **a**–**d** The mRNA and/or protein levels of AKT1, AKT2, p-AKT, c-Myc, STAT3, β-catenin, TGF-β, p-SMAD2, p-SMAD3, YAP and FOXO1 in Lenti-TCEAL7/si-TCEAL7-transfected WM-115 and A375 cells were determined by RT-PCR and western blotting assays. **e**–**g** Correlations between the expression levels of TCEAL7 and AKT1, AKT2 and c-Myc in melanoma samples were predicted by using the starBase database. **h**–**j**. Correlations between the expression levels of TCEAL7 and AKT1, AKT2 and c-Myc in 30 melanoma tissues samples were determined. (**a** and **c** *P < 0.05, compared with si-Scramble group; ^#^*P* < 0.05, compared with Lenti-NC group; **b** and **d**, *P < 0.05, compared with Lenti-NC group; ^#^*P* < 0.05, compared with si-Scramble group)

### TCEAL7 inhibits melanoma cell proliferation, migration and invasion through downregulating AKT1 and c-Myc

Then, we explored AKT1 and c-Myc roles in TCEAL7-mediated inhibition in melanoma progression. Compared with the lenti-TCEAL7 group, cell proliferation (Fig. 4a–d), invasion (Fig. 4e, f) and migration (Fig. 4i–l) abilities were significantly enhanced after the overexpression of either AKT1 or c-Myc in WM-115 and A375 cell lines, while cell apoptosis was reduced (Fig. 4g, h). These results demonstrated that TCEAL7 suppressed melanoma cell proliferation, migration and invasion through downregulating AKT1 and c-Myc.

**Fig. 4:** TCEAL7 inhibited the progression of melanoma through decreasing the expression of AKT1 and c-Myc. WM-115 and A375 cells were divided into Lenti-TCEAL7, Lenti-NC, Lenti-TCEAL7 + Lenti-AKT1/c-Myc and Lenti-AKT1/c-Myc groups and submitted to the following assays. **a**–**d** Cell proliferation was detected by using the CCK-8 assay. **e**, **f** Transwell chamber assay was used to detect cell invasion. **g**, **h** Flow cytometry assay was applied to detect cell apoptosis. **i**–**l** Scratch assay was used to assess cell migration ability. (*P < 0.05 and ***P < 0.001, compared with Lenti-NC group; ^#^*P* < 0.05 and ^###^*P* < 0.001, compared with Lenti-TCEAL7 group)

### MiR-758-3p downregulates TCEAL7 expression in melanoma cells

To further reveal the underlying mechanisms of TCEAL7 in melanoma progression, the databases of miRanda and miRDB were used to search the upstream miRNAs which target TCEAL7. The results showed that the co-regulator of TCEAL7 from both miRanda and miRDB databases was miR-758-3p (Fig. 5a). We then explored miR-758-3p expression levels in melanoma tissues and cells using RT-PCR assay. The results showed that miR-758-3p was upregulated in melanoma tissues and cell lines, A375 and WM-115 (Fig. 5b, c). The high expression level of miR-758-3p predicted a shorter overall survival time in patients with melanoma (Fig. 5d). In addition, miR-758-3p level showed a negative correlation with TCEAL7 level in melanoma tissues (Fig. 5e). Next, we explored miR-758-3p effect on the expression of TCEAL7. miR-758-3p level was significantly elevated when A375 and WM-115 cells were transfected with mimics-miR-758-3p as compared with the control group (Fig. 5f), which obviously reduced TCEAL7 level (Fig. 5g). Moreover, the luciferase gene reporter assay showed that the transcriptional activity of TCEAL7 was repressed following of miR-758-3p upregulation in A375 and WM-115 cells, whereas mutation of the binding sites between miR-758-3p and TCEAL7 3′UTR abrogated this effect (Fig. 5h–j). All of these results indicated that miR-758-3p was overexpressed in melanoma and negatively regulated TCEAL7 expression.

**Fig. 5:** miR-758-3p negatively modulated TCEAL7 expression. **a** BioVenn (https://www.biovenn.nl/index.php) was built to find the co-regulator of TCEAL7 from miRanda and miRDB diabetes. **b** RT-PCR analysis of the expression levels of miR-758-3p in melanoma tissues and nevus tissues (normal control). **c** RT-PCR was applied to determine miR-758-3p levels in normal melanocyte PIG1 and melanoma cell lines WM-115 and A375. **d** Kaplan–Meier was used to analyze the prognostic value of miR-758-3p in melanoma patients. **e** Correlation analysis between the expression levels of TCEAL7 and miR-758-3p in 30 melanoma tissues samples were determined. **f** RT-PCR analysis of the expression levels of miR-758-3p following cell infection with mimics-miR-758-3p or mimic-NC in WM-115 and A375 cells. **g** Western blotting analysis of the effect of miR-758-3p on the expression of TCEAL7 protein. **h** Putative binding sites between miR-758-3p and TCEAL7 3′UTR. **i**, **j** Dual-luciferase gene reporter system was used to assess the effect of miR-758-3p on the transcriptional activity of TCEAL7. (*P < 0.05, **P < 0.01, ***P < 0.001)

### miR-758-3p facilitates melanoma progression via inhibiting TCEAL7 expression

We next investigated whether miR-758-3p was involved in the progression of melanoma via targeting TCEAL7. CCK-8, transwell and starch assays results showed that cell proliferation (Fig. 6a, b), invasion (Fig. 6c) and migration (Fig. 6e, f) capacities were enhanced when WM-115 and A375 cells were infected with mimics-miR-758-3p, but these roles were impaired when TCEAL7 was overexpressed on the base of mimics-miR-758-3p treatment. In addition, cell apoptosis was inhibited when miR-758-3p was upregulated in WM-115 and A375 cells, and this role was impaired when cells were transfected with Lentiv-TCEAL7 on the base of mimics-miR-758-3p (Fig. 6d). Furthermore, animal assay was carried out in A375 cells to reveal miR-758-3p/TCEAL7 role in melanoma growth. The in vivo xenotransplantation assay showed that upregulation of TCEAL7 repressed the tumorigenesis of A375 cells, while miR-758-3p overexpression promoted tumor formation. In addition, TCEAL7 overexpression significantly abolished the pro-tumor effect of miR-758-3p (Fig. 7a, b). And, the expressions of miR-758-3p, AKT1, AKT2 and c-Myc were elevated, while TCEAL7 expression was decreased in tumor tissues in the mimics group, whereas this effect was impaired following TCEAL7 overexpression (Fig. 7c–e). Taken together, these above findings demonstrated that miR-758-3p facilitated melanoma progression by targeting TCEAL7.

**Fig. 6:** miR-758-3p promoted cell growth, migration and invasion and reduced cell apoptosis in melanoma via targeting TCEAL7. WM-115 and A375 cells were divided into mimic-NC + Lenti-NC, mimics + Lenti-NC and mimics + Lenti-TCEAL7 groups, and submitted to the following assays. **a**, **b** CCK-8 assay was used to test cell proliferation viability. **c** Transwell chamber assay was used to detect cell invasion. **d** Flow cytometry assay was applied to detect cell apoptosis. **e**, **f** Scratch assay was used to assess cell migration ability. (*P < *0.05*, compared with mimic-NC + Lenti-NC group; ^#^*P* < *0.05*, compared with mimics + Lenti-NC group)

**Fig. 7:** miR-758-3p promoted the tumorigenesis of melanoma cells via targeting TCEAL7. **a**, **b** In vivo tumor formation assay was carried out to detect the tumorigenesis in A375 cells from mimic-NC + Lenti-NC, mimics + Lenti-NC and mimics + Lenti-TCEAL7 groups. **c** RT-PCR analysis of the expression levels of miR-758-3p in tumor tissues. **d**, **e** RT-PCR and western blotting assays were applied to detect the mRNA and protein levels of TCEAL7, AKT1, AKT2 and c-Myc in tumor tissues. (*P < 0.05 and **P < 0.01, compared with mimic-NC + Lenti-NC group; ^#^*P* < *0.05*, compared with mimics + Lenti-NC group)

## Discussion

The malignant melanoma is characterized by aberrant proliferation, apoptosis reduction, and high motility and invasive potentials, which are of importance to maintain the aggressive clinical course [17, 18]. Herein, we explored the effects of TCEAL7 on cell proliferation, apoptosis, invasion, migration and tumorigenesis in melanoma, as well as uncovered the underlying mechanisms. The results showed that TCEAL7, negatively regulated by miR-758-3p, served as a tumor suppressor in melanoma through downregulating AKT1 and c-Myc.

TCEAL7 is a newly-identified pro-apoptotic protein that shares amino-acid sequence homology with the TCEAL1 (p21/SIIR/pp21) and the pp21 homolog (WBP5/TCEAL6) [4]. TCEAL7 was identified to be frequently downregulated in tumors as compared with the corresponding normal tissues, such as ovarian cancer, endometrial carcinoma and gastric adenocarcinoma [4, 6, 19]. The present study demonstrated, for the first time, that TCEAL7 was also lowly expressed in melanoma tissues and cell lines. In addition, we observed that low level of TCEAL7 was closely associated with shorter overall survival and advanced clinical features in melanoma patients, including larger tumor size, higher histological and TNM grades. Consistently, Huang et al. [6] reported that low expression level of TCEAL7 was closely correlated with larger tumor size, higher histological grade, lower survival and worse nodal status in gastric adenocarcinoma.

Increasing evidence has identified that TCEAL7 exerts a tumor-suppressive role. For instance, Chien et al. [4] reported that TCEAL7 induced cell death and inhibited cell colony formation efficiency in ovarian cancer cells. Guo et al. [19] found that TCEAL7 overexpression reduced cell proliferation and colony formation ability and downregulated the expression levels of the pro-proliferative genes, such as c-Myc and cyclin D1, and inhibited NF-κB activation. In the present study, we upregulated TCEAL7 in TCEAL7-null WM-115 cells, and both upregulate and downregulate TCEAL7 in A375 cells to study TCEAL7 role in melanoma progression. We found that TCEAL7 overexpression caused significant inhibitions in cell proliferation, invasion and tumorigenesis capacities and induced cell apoptosis in melanoma WM-115 and A375 cells, indicating that TCEAL7 serves as a tumor suppressor in melanoma.

In mechanism, we assessed the effects of TCEAL7 on the regulation of key signaling pathways. The results showed that TCEAL7 overexpression led to significant decreases in the expression levels of AKT1, AKT2 and c-Myc in WM-115 and A375 cells at both mRNA and protein levels. Further studies have shown that TCEAL7 level in melanoma samples showed significantly negative correlation with the expression levels AKT1 and c-Myc, but with no significant correlation with AKT2 level. Upregulation of either AKT1 or c-Myc abolished TCEAL7 roles in inhibiting cell proliferation, invasion and migration and inducing cell apoptosis in both A375 and WM-115 cells, indicating that TCEAL7 inhibited melanoma progression via decreasing AKT1 and c-Myc expression. Consistently, previous studies have revealed that TCEAL7 negatively regulated c-Myc expression in cancers [8, 20].

Through degrading mRNA of target genes, miRNAs serve important roles in tumor development and progression [21, 22]. It was previously reported that endogenous miR-182 degraded TCEAL7 mRNA and inhibited its translation [19]. With the help of bioinformatics analysis, TCEAL7 was predicted to be a target of miR-758-3p, which was verified by the luciferase gene reporter and western blotting assays. MiR-758-3p has been identified to be abnormally expressed and implicated in various kinds of cancers. For example, miRNA-758-3p expression was repressed by chemotherapy drugs in esophageal cancer [23]. MiR-758 was downregulated in papillary thyroid cancer [24], bladder cancer [25], glioblastoma [26], cervical cancer [27] and non-small cell lung cancer [28], and served as a tumor-suppressor. In the present study, we found that miR-758-3p was overexpressed in melanoma tissues and cells, and promoted cell growth, migration, invasion and tumorigenesis, and repressed the apoptosis of melanoma cells through downregulating TCEAL7 expression, indicating that miR-758-3p served as an oncogene in melanoma. We conjectured the different cancer types caused the difference in miR-758-3p roles in cancer progression. Evidence has demonstrated that the same miRNA may exert opposite roles in different types of cancers. For instance, miR-93-5p has been shown to promote cell proliferation in osteosarcoma [29], gliomas [30] and gastric cancer [31, 32], and enhance cell invasion ability in nasopharyngeal carcinoma [33]. In contrast, miR-93-5p suppresses cell invasion, migration and proliferation in breast cancer [34] and ovarian carcinoma [35].

## Conclusion

Collectively, our results showed that TCEAL7, regulated by miR-758-3p inhibited cell proliferation, migration, invasion and tumorigenesis and induced apoptosis in melanoma through downregulating AKT1, AKT2 and c-Myc levels (Fig. 8). Our study provides a potential therapeutic target (miR-758-3p/TCEAL7) for melanoma treatment.

**Fig. 8:** Schematic diagram of miR-758-3p/TCEAL7 in melanoma progression. TCEAL7, regulated by miR-758-3p inhibited cell proliferation, migration, invasion and tumorigenesis, and induced apoptosis in melanoma through downregulating AKT1, AKT2 and c-Myc expression levels

## Data Availability

All data generated or analysed during this study are included in this published article.

## Abbreviations

TCEAL: Transcription elongation factor A-like 7
3′UTR: 3′‑Untranslated regions
miRNAs: MicroRNAs
CCK-8: Cell Counting Kit-8
